The article "Electroacupuncture Synergistically Inhibits Proinflammatory Cytokine Production and Improves Cognitive Function in Rats with Cognitive Impairment due to Hepatic Encephalopathy through p38MAPK/STAT3 and TLR4/NF-κB Signaling Pathways" was published in 2021. Journal: Evid Based Complement Alternat Med.

# Electroacupuncture Synergistically Inhibits Proinflammatory Cytokine Production and Improves Cognitive Function in Rats with Cognitive Impairment due to Hepatic Encephalopathy through p38MAPK/STAT3 and TLR4/NF-*κ*B Signaling Pathways

**DOI:** 10.1155/2021/7992688

**Published:** 2021-10-01

**Authors:** Jiling Huang, Zhigang Gong, Yingnan Kong, Yanwen Huang, Hui Wang, Yingjie Kang, Songhua Zhan

**Affiliations:** Department of Radiology, Shuguang Hospital Affiliated to Shanghai University of Traditional Chinese Medicine, Shanghai 201203, China

## Abstract

**Objective:**

To investigate the effect of electroacupuncture (EA) on cognitive dysfunction in rats with hepatic encephalopathy and its underlying mechanism.

**Methods:**

Fifty Wistar rats were randomly divided into a normal group (*n* = 10) and model group (*n* = 40). Rat models of hepatic encephalopathy were established by administration of carbon tetrachloride and thioacetamide for a total of 12 weeks. At the 9th week after modeling, rats with cognitive impairment in the model group were identified by conducting the Morris water maze test, which were then randomly divided into a control group (CCl_4_) and treatment groups including EA group (CCl_4_ + EA), lactulose group (CCl_4_ + Lac), and EA plus lactulose group (CCl_4_ + CM), with 9 rats in each group. At the end of the 9th week, rats in CCl_4_ + Lac and CCl_4_ + CM groups had lactulose gavage at a dose of 10 mL/kg body weight, while normal control and CCl_4_ groups had gavage with the same volume of normal saline once a day for 21 days until the end of the experiment. Rats in CCl_4_ + EA and CCl_4_ + CM groups underwent acupuncture at Baihui (GV[DU]20), Shenting (GV[DU]24), and Zusanli (ST36) acupoints, among which EA at Baihui and Shenting acupoints were given once daily for 30 min lasting for 21 consecutive days. The effect of the treatment was measured by the Morris water maze test for learning and memory ability and magnetic resonance spectroscopy (MRS) for neuronal metabolism in the hippocampus of rats with hepatic encephalopathy. Pathological change in the rat hippocampus was observed by HE staining, while serum ammonia and liver function markers were detected. Western blot and real-time fluorescent quantitative PCR were used to detect the expressions of specific genes and proteins in the brain tissue.

**Results:**

Compared with those in the control group, rats undergoing EA had significantly shortened escape latency and increased number of platform crossing. H&E staining confirmed that EA improved brain tissue necrosis and ameliorated nuclear pyknosis in rats with hepatic encephalopathy. Significantly decreased levels of serum ammonia, alanine aminotransferase (ALT), aspartate transaminase (AST), total bilirubin (TBil), and total bile acid (TBA) were observed in rats undergoing EA, as well as improved levels of total protein (TP) and albumin (ALB). In addition, EA inhibited the brain expressions of TNF-*α*, IL-1*β*, IL-6, iNOS, TLR4, MyD88, NF-*κ*B, p38MAPK, phosphorylated (p)-p38MAPK, STAT3, and p-STAT3 genes, as well as protein expressions of TNF-*α*, IL-6, TLR4, MyD88, NF-*κ*B, p38MAPK, p-p38MAPK, STAT3, and p-STAT3. MRS showed increased Glx/Cr and decreased NAA/Cr, Cho/Cr and mI/Cr in the control group, and EA significantly reversed such changes in Glx/Cr and mI/Cr values.

The article "Electroacupuncture Synergistically Inhibits Proinflammatory Cytokine Production and Improves Cognitive Function in Rats with Cognitive Impairment due to Hepatic Encephalopathy through p38MAPK/STAT3 and TLR4/NF-κB Signaling Pathways" was published in 2021. Journal: Evid Based Complement Alternat Med.

**Conclusion:**

EA ameliorated the production of excessive proinflammatory cytokines in the hippocampus of rats with cognitive dysfunction secondary to hepatic encephalopathy, which also gave rise to subsequent changes such as reduced blood ammonia level, brain-protective activated astrocytes, and lower degree of brain tissue injury. The p38MAPK/STAT3 and TLR4/MyD88/NF-*κ*B signaling pathways may be involved. EA can also improve the metabolism of NAA and Cho in the rat hippocampus and thereby improve learning and memory abilities.

## 1. Introduction

Hepatic encephalopathy (HE), a central nervous system dysfunction due to metabolic disorders, is caused by acute and chronic liver dysfunction or portal-systemic shunt [1]. It is characterized by extensive neuropsychiatric changes, consciousness disorders, behavioral abnormalities, and a series of dysfunction ranging from subclinical changes to coma, which is a continuous process of neurocognitive dysfunction [2]. Among others, C-type HE (CHE) is the most common type that is associated with cirrhosis, portal hypertension, and/or portal shunt. Studies have shown that CHE is independently associated with death in patients with cirrhosis, and the onset of HE in such patients may lead to persistent and cumulative cognitive impairments [3], including brain dysfunction affecting learning, memory, attention, executive function, and reasoning. These impairments would directly compromise patients' activities of daily living and quality of life and thereby bring huge economic burden and serious social issues [4]. However, therapeutic strategy to effectively improve cognitive dysfunction in patients with hepatic encephalopathy after cirrhosis remains to be discovered.

The exact pathogenesis of HE remains unclear. Studies have investigated on the synergistic effect of ammonia and inflammation on astrocyte swelling and brain edema by inducing oxidative stress and mitochondrial damage with the involvement of other factors [5, 6]. Hyperammonemia can induce neutrophil dysfunction, release reactive oxygen species, and trigger oxidative stress and inflammation. In rat models with hyperammonemia, ammonia induced the activation of astrocytes and microglia in the hippocampus and release of brain-derived inflammatory factors such as iNOS, IL-1*β*, and TNF-*α*, thereby damaging cerebral endothelial cells and disrupting the blood-brain barrier. This will result in increased permeability, which would act synergistically with intestinal ammonia to aggravate neuroinflammation and brain edema, trigger neuroinflammation, and affect brain function [7, 8]. Furthermore, abnormalities in neurotransmitters such as glutamate can be initiated by altered expressions of corresponding receptors, which leads to cognitive impairment [9]. Relevant studies have shown that anti-inflammatory treatment can reduce portal vein pressure and improve cognitive function in mice by mitigating inflammatory cytokines [10]. As one of the important members of MAPK, p38MAPK plays a regulatory role in neuronal growth, brain tissue development, and cardiac cell growth [11]. Toll-1ike receptor 4 (TLR4) also plays an important role in inflammation as a transmembrane protein receptor that mediates innate immunity, which is associated with host cell recognition of various microbial pathogenic agents [12]. TLR4 specifically identifies pathogen-associated molecular patterns (PAMPs) and transmembrane signal transduction to deliver pathogen-associated molecular stimulus signals intracellularly and triggers a cascade of signals through myeloid differentiation factor 88 (MyD88). The inhibiting unit of nuclear factor kappa-B (NF-*κ*B), I*κ*B*α*, is subsequently phosphorylated and degraded, allowing NF-*κ*B and I*κ*B*α* to dissociate into the nucleus and bind specifically to *κ*B transcriptional regulation sequence located within the promoter or enhancer of downstream genes. As a result, the expression of inflammation-related genes would eventually lead to the release of various inflammatory cytokines and subsequent inflammatory responses [13].

The article "Electroacupuncture Synergistically Inhibits Proinflammatory Cytokine Production and Improves Cognitive Function in Rats with Cognitive Impairment due to Hepatic Encephalopathy through p38MAPK/STAT3 and TLR4/NF-κB Signaling Pathways" was published in 2021. Journal: Evid Based Complement Alternat Med.

The mainstay treatment for CHE is prompt removal of the precipitating factors and reversing the acute mental abnormality to a relatively stable state [14]. Lactulose is the first-line agent recommended in the current treatment guidelines for HE. Studies by Karakan et al. [15, 16] showed that lactulose can improve patients' cognitive function and reduce the incidence of symptomatic HE. However, the gastrointestinal adverse effects of lactulose have limited its usage, and it is not recommended for long-term clinical application due to its potential toxicity and the development of drug-resistant strains. Therefore, a safer and more effective treatment for HE is warranted. Acupuncture has been reported to play a regulatory role in the neuro-endocrine-immune network under stress. Mechanistically, acupuncture clears the meridians, regulates qi and the mind by stimulating the acupoints, and modulates the release of neurotransmitters and hormones in the neuro-endocrine-immune system. Thereby, it improves the ability of the body to cope with stress-related injury. Moreover, as a noninvasive alternative therapy, acupuncture can directly affect the nerve damage in the brain and improve cognitive dysfunction [17, 18]. However, the value and mechanism of acupuncture in the treatment of HE remain to be elucidated.

Magnetic resonance spectroscopy (MRS), a noninvasive approach to investigate the biochemical metabolic changes in the brain, reflects the concentration of compounds and metabolites in tissues and cells by utilizing the difference of hydrogen proton magnetic resonance frequency in different compounds and the height and area of the resonance peak [19]. MRS provides a new approach for early diagnosis and monitoring of HE by direct measurement of the concentration of osmotic substances such as mIns, Cho, and NAA. The hippocampus is an important functional region of the nervous system that is closely related to learning and memory. In this study, by observing the effect of electroacupuncture (EA) on the production of inflammatory factors such as IL-1*β*, TNF-*α*, and IL-6 in rats with cognitive impairment in CHE, we explored the role of TLR4/MyD88/NF-*κ*B and p38MAPK/STAT3 signaling pathways in improving CHE-related cognitive impairment in rats undergoing EA, as well as the underlying mechanism and therapeutic targets.

## 2. Materials and Methods

### 2.1. Main Instruments and Reagents

The aspartate aminotransferase (AST) test kit (batch number: 01ast180109), alanine aminotransferase (ALT) test kit (batch number: 01ast180108), and total bile acid (TBA) test kit (batch number: 2401698) were purchased from Shanghai Huachen Bearing Technology Co., Ltd. (Shanghai, China). The total bilirubin (TBil) test kit (Lot: 180824101), total protein (TP) test kit (Lot: 2401106), and serum albumin (ALB) test kit (Lot: 2400122) were purchased from Medical System Biotechnology Co., Ltd. (Ningbo, China). Carbon tetrachloride (CCl_4_) (batch number: 89106125), thioacetamide (TAA) (batch number: 20160930), and olive oil (batch number: c10728873) were purchased from Shanghai Chemical Industry Park (Shanghai, China); lactulose (batch number: h20103621) made by Sichuan Jianneng Pharmaceutical Co., Ltd. The hematoxylin and eosin (H&E) staining test kit (batch number: 20180720) and blood ammonia assay kit (batch number: 2400505) were purchased from Nanjing Jiancheng Bioengineering Institute (Nanjing, China). TNF-*α* (60291-1-Ig), IL-1*β* (12703), IL-6 (12153), TLR4 (14358), MYD88 (4283), NF-*κ*B (8242), p38MAPK (6417), (p)-p38MAPK (8690), STAT3 (9139), p-STAT3 (9145), and INOS (SBJ_M0506) were purchased from Cell Signaling Technology. Special fixation frames for rat acupuncture experiment (purchased from Beijing Global Biotechnology Co., Ltd.), 0.18 mm*∗*13 mm acupuncture needles (batch number: 20071723; Beijing Zhongyan Taihe Medical Instrument Co., Ltd.), the Huatuo SDZ-V pulse acupuncture therapy instrument (Shanghai Huayi Medical Instrument Co., Ltd.), and the Siemens Skyra 3.0T scanner were used for magnetic resonance spectroscopy. Digbehv animal behavior analysis system includes Morris water maze, computer camera system, and software analysis system, purchased by Shanghai Jilu Software Technology Co., Ltd.

The article "Electroacupuncture Synergistically Inhibits Proinflammatory Cytokine Production and Improves Cognitive Function in Rats with Cognitive Impairment due to Hepatic Encephalopathy through p38MAPK/STAT3 and TLR4/NF-κB Signaling Pathways" was published in 2021. Journal: Evid Based Complement Alternat Med.

### 2.2. Experimental Animals and Modeling Methods

50 Wistar male rats (200 ± 20 g, SPF grade)—provided by the Experimental Animal Center of Shanghai University of Traditional Chinese Medicine under animal license number SYXK (Shanghai, 2020-0009) and ethics committee document No.: PZSHUCM200703001—were maintained at an animal facility under pathogen-free conditions. The handling of rats and experimental procedures were conducted in accordance with experimental animal guidelines. Rat models with cirrhosis were established according to a previously reported protocol by Matei et al. [20, 21]. Fifty Wistar rats were randomly divided into a normal control group (*n* = 10) and model group (*n* = 40) according to the weight stratification method after adaptive feeding for one week. The HE model was established with carbon tetrachloride combined and thioacetamide (TAA) for 9 weeks. The model group was intraperitoneally injected with 1 mL/kg 35% carbon tetrachloride (diluted with olive oil) twice a week. At the end of the 9th week, TAA (3.5%, 250 mg/kg) was injected daily for 2 days in each group. After TAA injection in rats, the presence of any one of the symptoms such as drowsiness, slow reaction, reduced voluntary activity, ataxia, and coma can be diagnosed as HE. Before modeling, all rats were subjected to the Morris water maze test. At the 9th week after modeling, rats with cognitive impairment were screened through the Morris water maze test and randomly divided into a no-intervention group (CCl_4_) and treatment groups including EA group (CCl4 + EA), lactulose group (CCl4 + Lac), and EA combined with lactulose group (CCl_4_ + CM), with 9 rats in each group. Among them, therapeutic interventions were given in CCl4 + EA, CCl_4_ + Lac, and CCl_4_ + CM groups, which were regarded as interventional groups. At the end of the 9th week, the CCl_4_ + Lac group and the CCl_4_ + CM group were gavaged with lactulose at a dose of 10 mL/kg body weight, while normal control and CCl_4_ groups were gavaged with the same volume of normal saline once a day for 21 days until the end of the experiment. All rats were fed with common fodder and had free intake of food and water during the study period. Finally, at the end of the 12th week of intervention, the rats' learning and memory function was measured by using the Morris water maze.

The article "Electroacupuncture Synergistically Inhibits Proinflammatory Cytokine Production and Improves Cognitive Function in Rats with Cognitive Impairment due to Hepatic Encephalopathy through p38MAPK/STAT3 and TLR4/NF-κB Signaling Pathways" was published in 2021. Journal: Evid Based Complement Alternat Med.

### 2.3. EA Treatment

At the end of week 9, EA was given to rats in the CCl_4_ + EA and CCl_4_ + CM groups. Rats were placed in a dedicated fixative for rat acupuncture and moxibustion, and acupoint selection was done by referring to the textbook of *experimental acupuncture* [22]. The skin areas of “Housanli” on both sides (equivalent to “Zusanli” point), “Baihui”, and “Shenting” acupoints were disinfected with 75% ethanol. The acupoints were then treated with disposable sterile acupuncture needles (0.18 × 13 mm), and each point was twisted and supplemented for 1 min. The needle penetration depth is about 4 mm, which indicates the Deqi of acupuncture. Electric stimulation at “Baihui” and “Shenting” was conducted by using a Hwato EA therapeutic instrument with a frequency of 10 Hz and an intensity of 1 to 2 mA (continuous wave). The positive pole is connected to the Baihui point, and the negative pole is connected to the Shenting point, forming a loop. The appearance of slight tremor of rat limbs along with the frequency of EA apparatus was regarded as a sign of appropriate intensity. Each EA stimulus lasted for 30 min and was given once daily for consecutive 21 days.

### 2.4. Morris Water Maze Experiment

The Morris water maze test was used to measure the learning and memory ability of rats in each group before and after modeling and after treatment with EA. A black round pool with a diameter of about 150 cm and a height of about 60 cm was used, and the cross was divided into four quadrants, namely upper left, upper right, lower left, and lower right. A circular transparent platform with a diameter of about 12 cm was placed in the center of the upper right quadrant, and the position and size of the platform were recorded as the target area. Water was put into the pool at a height of about 2 cm higher than the platform, and the water temperature was adjusted to 25 ± 1 °C. The water in the pool was stained with carbon ink so that the rats could not see the location of the platform. All water maze experiments were carried out in the morning for 4 consecutive days. Directional sailing test: Rats were put into the water from any quadrant facing the markers each time and allowed to swim freely to find the platform under the water surface for 60 s. If the rats climbed to the platform within 60 s, this period was recorded as latency. The incubation period was 60 s, and the rats were artificially guided to the platform to rest for 20 s. The same procedure was done in all four quadrants. Space exploration experiment: After the directional navigation test for 3 days, the cylindrical platform was removed and the rats were put into water. The computer automatic monitoring system tracked and recorded the number of times that the rats passed through the original platform position within 90 s, and the mean value of each group was taken for observation and comparative analysis. The escape latency and times of crossing the platform on the fourth day were used to assess the learning ability and memory of the rats.

The article "Electroacupuncture Synergistically Inhibits Proinflammatory Cytokine Production and Improves Cognitive Function in Rats with Cognitive Impairment due to Hepatic Encephalopathy through p38MAPK/STAT3 and TLR4/NF-κB Signaling Pathways" was published in 2021. Journal: Evid Based Complement Alternat Med.

### 2.5. MRI Examination

MRI was performed at the end of the third Morris water maze test. The Siemens 3.0T Skyra MRI scanner with special coil for rats (Shanghai Guangcheng Company; model CG-MUC40-H300-AS) was utilized for MRI imaging of rats. After anesthesia with intraperitoneal 3% pentobarbital at a dose of 2 mL/kg, the rats were placed in the coil with the prone position so that the brain was located in the middle part of the coil. After conventional transverse and coronal T2WI and T1WI MRI scanning, 1H-MRS scanning was performed [23]. Using single voxel spectroscopy (SVS)-stimulated echo acquisition mode spectroscopy (STEAM), the brain was scanned by 1H-MRS with TR/TE = 2000/9.53 ms and a turn angle of 90°. The mean acquisition time was 128, the scanning time was 4 minutes and 25 seconds, and the voxel size was 1*∗*1*∗*1 cm. Scan was localized in the hippocampus of the rat brain, and the skull was avoided. Shimming was carried out in the VOI with the full width at half maximum of the water peak less than 8 Hz. Meanwhile, the resonance frequency of water was determined and input into the chemical shift selection sequence. The optimal water suppression effect was obtained by adjusting pulse excitation angle in the sequence.

After scanning, the baseline calibration, signal averaging, metabolite identification, and calculation of the area under the peak curve of metabolites were completed with the software attached to the device. The positions of the chemical shift of the metabolites were as follows: N-acetylaspartic acid (NAA): 2.01 ppm; alkali complex (Cho): 3.22 ppm; inositol (mI): 3.22 ppm; peak of creatinine (Cr): 3.03 ppm; glutamic acid-glutamine complex (Glx): 3.75 ppm. The ratios of the areas under the curve of each metabolite—i.e., NAA/Cr, CHO/Cr, MI/Cr, and GLX/Cr—were calculated with creatine (Cr) as the reference.

The article "Electroacupuncture Synergistically Inhibits Proinflammatory Cytokine Production and Improves Cognitive Function in Rats with Cognitive Impairment due to Hepatic Encephalopathy through p38MAPK/STAT3 and TLR4/NF-κB Signaling Pathways" was published in 2021. Journal: Evid Based Complement Alternat Med.

### 2.6. Sample Collection and Processing

After the MRS scan, craniotomy was performed under general anesthesia. The left brain was implanted with 10% formalin for fixation, and the right brain was separated from the hippocampus on a cryopreservation table. The hippocampus was placed in liquid nitrogen in a cryopreservation tube and stored at −80°C. Sampled brain tissues were dehydrated, embedded, and sliced before stained with H&E staining. Pathological changes of brain tissues were observed under a microscope. Blood sample was collected from the abdominal aorta, and part of the blood was treated with heparin sodium as an anticoagulant. The blood ammonia level was detected within 0.5 h. The remaining blood sample was placed at 4°C for 3 h before centrifugation at 3000 r/min for 15 min, and serum was obtained and stored at −70°C for later use.

### 2.7. Observation Index and Inspection Method

#### 2.7.1. Serum Biochemistry Assays

Rats were anesthetized with pentobarbital, and blood was collected from the abdominal aorta. The levels of serum ammonia, serum TBil, ALT, AST, TBA, TP, and ALB were measured in accordance with the kit instructions of Nanjing Jiancheng Bioengineering Institute.

#### 2.7.2. Evaluation of Brain Injury and Pathology

Brain tissues were fixed in 10% neutral-buffered formalin and embedded in paraffin. Sections of 5 *μ*m thickness were affixed to slides, deparaffinized, and stained with hematoxylin/eosin to observe the histological changes of the hippocampal CA1 region, whether there is cell necrosis or neuronal degeneration.

#### 2.7.3. Real-Time PCR

Real-time reverse transcription polymerase chain reaction (RT-PCR) primers were designed and synthesized by Shanghai Sangon Biological Engineering (Shanghai, China). Primers of TNF-*α*, IL-1*β*, IL-6, iNOS, TLR4, MyD88, NF-*κ*B, P38MAPK, and STAT3 mRNAs were designed and synthesized by BioTNT (Shanghai, China). Information of the aforementioned genes and their primer sequences are shown in Table 1. Total RNA was extracted from tissues using an RNA extraction kit (MagExtractor) according to the manufacturer's instructions; and the RNA concentration detector was corrected before 5 *μ*L of each sample was taken, and NanoDrop 2000 was used to detect the concentration and purity of RNAs. Extracted total RNAs were reverse-transcribed using reverse transcriptase kits according to the manufacturer's instructions. Using cDNA as a template, amplification was conducted using 10 *μ*L of SYBR Green qPCR mix system according to the instructions of the TOYOBO amplification kit.

#### 2.7.4. Western Blot Assay

Brain tissue (25 *μ*g) was added to an appropriate volume of RIPA (including protease inhibitor and phosphatase inhibitor) and let stand for 10 min before centrifuged at 12000 rpm, 4°C for 20 min, and the supernatant was collected. Protein concentrations were measured, and samples were prepared using the loading buffer. SDS-PAGE electrophoresis was done at 300 mA with constant flow, and a blocking solution was applied for 30 min. Primary antibodies were added and incubated overnight at 4°C. Primary antibodies were IL-6 (1:1000), iNOS (1 : 1000), p-p38 (1 : 1000), p38 (1 : 1000), TLR4 (1 : 1000), MyD88 (1 : 1000), NF-*κ*B (1:1000), TNF-*α* (1 : 1000), IL-1*β* (1 : 1000), STAT3 (1 : 1000), and p-STAT3 (1 : 1000). The product was washed with PBST for 3 times, each lasting for 5 min. The secondary antibody (1 : 3000) was then added and incubated at room temperature for 1 h before being washed with PBST. The PVDF membrane was placed on the image scanner, covered with chromographic solution, and reacted for 1–2 min. Discoloration was done with Photoshop software, and densitometric values of target bands were analyzed with the alpha software processing system. *β*-Actin was used as an internal reference, and the relative expression of the protein of interest was calculated as the ratio of the gray value of the protein of interest to the gray value of the internal reference.

The article "Electroacupuncture Synergistically Inhibits Proinflammatory Cytokine Production and Improves Cognitive Function in Rats with Cognitive Impairment due to Hepatic Encephalopathy through p38MAPK/STAT3 and TLR4/NF-κB Signaling Pathways" was published in 2021. Journal: Evid Based Complement Alternat Med.

### 2.8. Statistical Analysis

Statistical analysis was performed using IBM SPSS software, version 22.0 (Armonk, NY). Measurement data were expressed as mean ± standard deviation (*x* ± *s*). One-way ANOVA was used for comparison among multiple groups, and the LSD-*t* test was used for post hoc analysis. *P* ≤ 0.05 was considered statistically significant.

## 3. Results

### 3.1. EA Significantly Shortened the Escape Latency and Increased the Number of Platform Crossing

Morris water maze is a classic method to observe the spatial learning and memory abilities in experimental rodent models, in which animals are trained to navigate to a platform located below the water's surface for the spatial cognition test. In this study, no significant difference was found in the latency of water maze escape and the number of platform crossing (*P* > 0.05) in rats before HE modeling. After modeling, the escape latency in rats in the CCl_4_ group and treatment groups was significantly prolonged (*P* < 0.05), while the number of platform crossing was decreased (*P* < 0.05). No significant difference was found among the four groups (*P* > 0.05). After intervention, the escape latency in the CCl_4_ group was significantly prolonged (*P* < 0.05) compared with the normal group; contrarily, compared with the CCl_4_ group, the escape latency in CCl_4_ + EA, CCl_4_ + LAC, and CCl_4_ + CM groups was significantly shortened (*P* < 0.05) and the number of platform crossing was increased (*P* < 0.05), and the CCl_4_ + CM group was the most significant, as shown in Figure 1. The above results showed that EA improved the learning and memory disorders caused by HE.

The article "Electroacupuncture Synergistically Inhibits Proinflammatory Cytokine Production and Improves Cognitive Function in Rats with Cognitive Impairment due to Hepatic Encephalopathy through p38MAPK/STAT3 and TLR4/NF-κB Signaling Pathways" was published in 2021. Journal: Evid Based Complement Alternat Med.

### 3.2. EA Can Reduce Serum Ammonia Value and Significantly Improve Liver Function in Rats with HE

The disorder of blood ammonia metabolism is an important pathogenetic factor of HE. Alanine aminotransferase (ALT), aspartate transaminase (AST), albumin (ALB), total protein (TP), albumin (ALB), and total bilirubin (TBil) are commonly used indicators for liver function. These indicators can effectively reflect the inflammatory state of the liver and the degree of hepatocyte injury. Compared with normal control, serum levels of TBil, ALT, AST, and TBA in the CCl_4_ group were significantly increased (*P* < 0.001), and the levels of TP and ALB were significantly decreased (*P* < 0.05). Meanwhile, compared with the CCl_4_ group, the levels of TBil, ALT, AST, and TBA in CCl_4_+EA, CCl_4_+Lac, and CCl_4_+CM groups were significantly decreased (*P* < 0.05) and the TP level was significantly increased (*P* < 0.05), whereas the ALB level in the CCl_4_ + CM group was significantly increased (*P* < 0.05). Compared with the CCl_4_ group, AST levels in both CCl_4_ + EA and CCl_4_ + CM groups were significantly decreased (*P* < 0.05), while TBil and ALT levels in the CCl_4_ + CM group were significantly decreased (*P* < 0.05) (Figures 2(a)–2(f)). Compared with the normal group, the blood ammonia level in the CCl_4_ group was significantly increased (*P* < 0.01). Compared with the CCl_4_ group, blood ammonia content in CCl_4_ + EA, CCl_4_ + Lac, and CCl_4_ + CM groups was significantly decreased on average (*P* < 0.01), and the CCl_4_ + CM group was the most significant (Figure 2(g)). These results indicate that EA can significantly improve the liver function of rats with hepatic encephalopathy and improve brain edema by reducing blood ammonia.

### 3.3. EA Improved Rat Brain Injury Induced by CCl_4_ and TAA

HE staining of the brain tissues in the CA1 region of the hippocampus in rats of the normal group showed intact structure and normal size of neuron cells with absence of abnormal cells; while brain tissues in rats in the CCl_4_ group presented with prominent necrosis with irregular nuclear morphology, disrupted cell membrane, decreased cytoplasm volume, condensed chromatin with cytoplasmic dispersion, pyknosis, and neuronal axonal disorganization. Compared with those in the CCl_4_ group, rats in CCl_4_ + EA, CCl_4_ + Lac, and CCl_4_ + CM groups had significantly improved brain structure, especially in the CCl_4_ + CM group (Figure 3).

The article "Electroacupuncture Synergistically Inhibits Proinflammatory Cytokine Production and Improves Cognitive Function in Rats with Cognitive Impairment due to Hepatic Encephalopathy through p38MAPK/STAT3 and TLR4/NF-κB Signaling Pathways" was published in 2021. Journal: Evid Based Complement Alternat Med.

There are 10 rats in the normal group and 9 rats in each of no-intervention group (CCl_4_) and treatment groups including EA group (CCl4 + EA), lactulose group (CCl4 + Lac), and EA combined with lactulose (CCl_4_ + CM) group. H&E staining was used to evaluate the degree of brain inflammation. H&E (×200) staining.

### 3.4. EA Improved Nerve Cell Metabolism in the Hippocampus in Rats with Hepatic Encephalopathy

MRS was utilized for quantitative measurement of the changes in brain metabolites. Compared with the normal group, increased Glx/Cr values and decreased NAA/Cr, Cho/Cr, and mI/Cr values (all *P* < 0.05) were observed in the CCl_4_ group. After intervention, we found decreased Glx/Cr values and increased Cho/Cr and mI/Cr values in all treatment groups (all *P* < 0.05), especially in the CCl_4_ + EA group and CCl_4_ + CM group (*P* < 0.05) (Figure 4). The results suggest that EA combined with other treatments may be able to modulate the metabolism of NAA, Glx, and Cho in the hippocampus in rats with HE and thereby improve the learning and memory performance in Morris water maze.

### 3.5. EA Effectively Ameliorated Inflammation in HE Rats by Inhibiting Inflammatory Factors Such as TNF-*α*, IL-6, and IL-1*β*

Inflammation can aggravate cognitive impairment in conjunction with ammonia. In this study, mRNA and protein expressions of TNF-*α*, IL-1*β*, and IL-6 in brain tissues of rats in the CCl_4_ group were significantly upregulated compared with the normal control group (*P* < 0.01); Meanwhile, compared with the CCl_4_ group, the mRNA and protein expressions of TNF-*α*, IL-1*β*, and IL-6 in brain tissues of rats in each treatment group were significantly downregulated (*P* < 0.05), especially those in CCl_4_ + EA and CCl_4_ + CM groups (*P* < 0.05) (Figures 5(a)–5(c), 6(a), 6(b), 7(a)). Therefore, it is suggested that EA inhibits the inflammatory reaction in the brain by reversing the imbalance between anti-inflammatory and inflammatory factors.

Liver failure can lead to toxin accumulation, elevated blood ammonia level, and secondary brain dysfunction [24]. Elevated blood ammonia can stimulate iNOS expression, promote NO production, increase cerebral blood flow, and result in astrocyte edema. Rats in the CCl_4_ group had significantly increased expression of iNOS mRNA (vs normal group, *P* < 0.01). Meanwhile, rats in each treatment group had downregulated expression of iNOS mRNA in brain tissues (vs CCl_4_ group, *P* < 0.05); among which, rats in CCl_4_ + EA and CCl_4_ + CM groups had significantly decreased iNOS mRNA compared with the CCl_4_ + Lac group (*P* < 0.05) (Figure 5(d)).

The article "Electroacupuncture Synergistically Inhibits Proinflammatory Cytokine Production and Improves Cognitive Function in Rats with Cognitive Impairment due to Hepatic Encephalopathy through p38MAPK/STAT3 and TLR4/NF-κB Signaling Pathways" was published in 2021. Journal: Evid Based Complement Alternat Med.

### 3.6. EA Activated TLR4/MyD88/NF-*κ*B Signaling Pathway

The TLR4/MyD88/NF-*κ*B signaling pathway was widely distributed in various tissues and cells of the body, which can mediate the expression of inflammatory factors in cells [25]. Intervention of various targets in the TLR4/MyD88/NF-*κ*B signaling transduction pathway has been found to reduce the inflammatory response of tissue to brain injury [26]. Our results showed that compared with normal control, the mRNA and protein expressions of TLR4, MyD88, and NF-*κ*B in rat brains in the CCl_4_ group were significantly increased (all *P* < 0.001), while expressions of those in the brain of HE rats were significantly decreased (all *P* < 0.05). Moreover, mRNA and protein expressions of TLR4, MyD88, and NF-*κ*B in the CCl_4_ + CM group were significantly decreased compared with the CCl_4_+Lac group (*P* < 0.05) (Figures 5(e)–5(g), 6(c)–6(e), Figure 7(b)). Our results suggest that EA may alleviate brain injury in rats with HE by regulating the TLR4/MyD88/NF-*κ*B signaling pathway.

### 3.7. EA Inhibited the p38MAPK/STAT3 Signaling Pathway and Thereby Reduced the Inflammatory Response

As an important member of the mitogen-activated protein kinase family, the p38MAPK signaling pathway plays an essential role in inflammatory response and cell apoptosis. STAT3 is considered one of the possible substrates of MAPK, which is the common pathway of intracellular signal transmission among different inflammatory cells and various inflammatory mediators and is involved in various biological reactions such as immune response and cell proliferation, differentiation, migration, and apoptosis [27]. In this study, after 3 weeks of acupuncture treatment, the mRNA and protein expressions of p38MAPK, p-p38MAPK, STAT3, and p-STAT3 in brain tissues of rats in the CCl_4_ group were significantly increased compared with those in the normal control group (*P* < 0.001), indicating that MAPK and STAT3 signaling pathways could have simultaneously been activated under the inflammatory response in HE. Compared with the CCl_4_ group, the mRNA and protein expressions of p38MAPK, p-p38MAPK, STAT3, and p-STAT3 in brain tissues of HE rats in all treatment groups were significantly decreased (*P* < 0.05). Compared with the CCl_4_ + Lac group, expressions of p38MAPK, p-p38MAPK, STAT3, and p-STAT3 in the CCl_4_ + CM group were significantly downregulated (*P* < 0.05). No significant difference in mRNA and protein expression levels between CCl4 + EA and CCl_4_ + Lac groups (*P* > 0.05) was found (Figures 5(h), 5(i), 6(f)–6(i), 7(c)). In summary, EA downregulated the expressions of p38MAPK-STAT3 mRNA and related proteins by activating the p38MAPK-STAT3 signaling pathway and thereby modulated the inflammatory response in rats with HE.

The article "Electroacupuncture Synergistically Inhibits Proinflammatory Cytokine Production and Improves Cognitive Function in Rats with Cognitive Impairment due to Hepatic Encephalopathy through p38MAPK/STAT3 and TLR4/NF-κB Signaling Pathways" was published in 2021. Journal: Evid Based Complement Alternat Med.

## 4. Discussion

Currently, the pathogenesis of HE remains unclear, possible theories include toxication derived from excessive ammonia, *γ*-aminobutyric acid, manganese ions, and pseudo neurotransmitters, as well as oxidative stress and imbalance of serum amino acid [1]. Ammonia poisoning is the mainstay theory, and reducing the blood ammonia level serves as an important therapeutic strategy in the treatment of HE. A prospective clinical study has revealed a dose-dependent relationship between serum ammonia and cognitive dysfunction [28]. Studies on the effects of ammonia toxication on the pathogenesis of HE and neurological damage have made some progress. A study [29] investigating chronic HE in rats found that reduced blood ammonia could affect the expressions of liver function biomarkers, inflammatory factors, apoptotic genes, and neurotransmitters. Recently, the synergistic effect of blood ammonia and inflammatory mediators on the initiation and development of HE has drawn more attention [30]. Acupuncture, as one of the classic therapeutic modalities in traditional Chinese medicine, has its unique advantages such as multitarget, multilevel, and omnidirectional treatment approaches. Acupuncture can deliver therapeutic effects by stimulating the internal potential of the body through activation of various regulatory mechanisms. Modern studies have shown that acupuncture at specific acupoints can play a therapeutic role in HE via inhibition of inflammatory response, improvement in liver function, and reduction of the blood ammonia level [31]. In addition, through observation of hippocampal neuron morphology and brain-derived neurotrophic factors in rats under chronic stress state, a study reported that acupuncture improved the damage of central neurons under stress state and had a benign regulatory effect on brain-derived neurotrophic factors [32]. However, few studies have investigated the specific mechanism of acupuncture therapy in mitigating HE-related cognitive dysfunction. The “Zusanli” acupoint chosen in this study is one of the most commonly adopted acupoints in current studies on the treatment of liver diseases [33]. Additionally, Baihui and Shenting acupoints belong to Du meridian, which is thought to bear the mind-awakening effect. Preliminary clinical and preclinical studies have demonstrated the efficacy of acupuncture at Baihui and Shenting acupoints in the treatment of cognitive dysfunction [34]. Therefore, these three acupoints were selected for rat experiments in this study.

The article "Electroacupuncture Synergistically Inhibits Proinflammatory Cytokine Production and Improves Cognitive Function in Rats with Cognitive Impairment due to Hepatic Encephalopathy through p38MAPK/STAT3 and TLR4/NF-κB Signaling Pathways" was published in 2021. Journal: Evid Based Complement Alternat Med.

We used Morris water maze to investigate the spatial learning and memory of rats with HE-related cognitive impairment. It is a well-established approach used to test cognitive impairment, especially learning dysfunction in rats. The escape latency period and the number of platform crossing were selected to reflect the cognitive changes. We found shortened escape latency and increased number of platform crossing after EA treatment for 3 weeks in rats in CCl_4_ + Lac, CCl_4_ + EA, and CCl_4_ + CM groups, which indicates that EA can refresh the brain and resuscitate, regulate qi activity, relax tendons and activate collaterals, and promote the recovery of damaged brain tissue in rats, thus mitigating the learning and memory disturbances in rats with HE-related cognitive impairment.

The MRS technology uses the difference of hydrogen proton magnetic resonance frequency in different compounds and the peak height and area of the resonance peak to reflect the compound concentration, as well as the metabolism within tissues and cells, which can be used as an indicator for the early diagnosis of HE [35]. The metabolites commonly studied include N-acetylaspartate (NAA), creatine (Cr) and choline complex (Cho), glutamine and glutamate complex (Glx), myo-inositol (mIns), etc. Each metabolite is sensitive to different pathological processes. NAA peak mainly exists in neurons, which can reflect the density and functional state of neurons. Cho peak is a marker of cell membrane damage and glial cell proliferation and is a precursor of acetylcholine, an important neurotransmitter [36]. The peak of mIns is a marker of glial cells, and the abnormal changes of Cho and mI peaks indirectly reflect the changes in osmotic pressure inside and outside astrocytes. Glu is the most abundant amino acid in the brain and a major neurotransmitter. Glx composite peaks are mainly derived from the overlapping formants of glutamine (Gln) and glutamic acid (Glu) [37]. Since the level of Cr in the brain remains relatively stable, Cr is used as an internal parameter to quantify the levels of Glx, mIns, Cho, and NAA. Typical changes in patients with HE are decreased mI/Cr and Cho/Cr, increased Glx/Cr, and insignificant changes in NAA and NAA/Cr [38]. In this study, we found that compared with the normal group, mI/Cr, NAA/Cr, and Cho/Cr decreased and Glx/Cr increased in the HE model group, which was consistent with previous research results and also echoed the ammonia poisoning theory in HE. The underlying mechanism may be that liver dysfunction in HE patients may lead to hyperammonemia, which increases the blood ammonia concentration and damages the blood-brain barrier, thereby increasing glutamine synthesis in astrocytes and consequently increasing Glx peak. Elevated osmotic pressure in the brain leads to swelling of neurons, causing brain edema and further cognitive dysfunction [39]. Therefore, the elevation of Glx/Cr is closely related to the severity of HE. Meanwhile, the production of glutamine increases the osmotic pressure in astrocytes, and cells compensate for the high osmotic pressure by expulsing osmotic agents such as Mi and Cho, resulting in decreases in mI/Cr and Cho/Cr ratios. However, the NAA/Cr value in rats in the CCl_4_ group was found to be decreased in this study, indicating an advanced-stage HE and impaired neuronal function. These results further validated the success of the HE rat model and reflected that the changes in brain metabolites had certain diagnostic value in HE. After 3 weeks of EA treatment, Glx/Cr, NAA/Cr, Cho/Cr, and mI/Cr were significantly decreased in the CCl_4_ + EA group, while the levels of NAA/Cr, Cho/Cr, and mI/Cr were significantly increased compared with the CCl_4_ group. Compared with the CCl_4_ + Lac group, the CCl_4_ + EA group has no significant difference, while the CCl_4_ + CM group has the most significant effect. These results indicate that abnormal brain metabolism shown by MRS is reversible, and EA may protect neurons and improve cognitive function by regulating the metabolism of NAA, Glx, and Cho in rats with HE.

The article "Electroacupuncture Synergistically Inhibits Proinflammatory Cytokine Production and Improves Cognitive Function in Rats with Cognitive Impairment due to Hepatic Encephalopathy through p38MAPK/STAT3 and TLR4/NF-κB Signaling Pathways" was published in 2021. Journal: Evid Based Complement Alternat Med.

Inflammatory response contributes to the pathological changes of HE to a large extent. A recent study [40] has confirmed that immune inflammatory response is involved in the occurrence and development of cognitive dysfunction. Inflammatory cytokines such as TNF-*α*, IL-1*β*, and IL-6 are main contributors for pathophysiological processes via maintaining chronic inflammatory state and inducing inflammatory cascade amplification. TNF-*α* induces the production of “secondary” cytokines such as IL-1*β* and IL-6 in the inflammatory response and thereby stimulates cytokine cascade reaction and inflammatory chain reaction. Studies have revealed a strong correlation between TNF-*α* level and HE, thus indicating that TNF-*α* can be used as a predictor of HE severity [41]. IL-6, also known as a proinflammatory factor, can activate microglia and astrocytes and cause neuronal damage and cognitive impairment by inducing the production of neurotoxic transmitters. Although inflammatory cytokines such as TNF-*α*, IL-1*β*, and IL-6 cannot directly penetrate the blood-brain barrier, they can damage the permeability of the blood-brain barrier to a certain extent. Meanwhile, active transport of substances to the brain could lead to swelling of astrocytes and inflammatory reactions in the brain. Impairment of liver function causes hyperammonemia, in which blood ammonia concentration increases and hampers the blood-brain barrier before entering the brain tissue. Increased osmotic pressure in the brain leads to swelling of neuronal cells, causing brain edema, which synergistically promotes the development of HE. Therefore, effective antagonization of TNF-*α*, IL-1*β*, and IL-6 could be a therapeutic strategy to mitigate hepatic encephalopathy.

The article "Electroacupuncture Synergistically Inhibits Proinflammatory Cytokine Production and Improves Cognitive Function in Rats with Cognitive Impairment due to Hepatic Encephalopathy through p38MAPK/STAT3 and TLR4/NF-κB Signaling Pathways" was published in 2021. Journal: Evid Based Complement Alternat Med.

Inflammatory response can be mediated by a variety of signaling pathways, among which TLR4/MyD88/NF-*κ*B is one of the mainstay pathways mediating inflammatory reactions all over the body. In the central nervous system, TLR4 is mainly expressed in glial cells. Studies have demonstrated the relationship between TLR4 expression and blood ammonia level and found that the inhibition of TLR4 expression in rats can alleviate blood ammonia release, thereby preventing HE [42]. NF-*κ*B is a protein complex widely involved in biological processes such as inflammation, apoptosis, immune response, and cell growth and development. During macrophage activation, upstream TLR4 triggers intracellular signal transduction, which ultimately activates NF-*κ*B through stimulating MyD88 [43]. NF-*κ*B activation can further trigger the release of inflammatory cytokines such as TNF-*α*, IL-1*β*, and IL-6 [44]. Consistently, TAA-induced NF-*κ*B expression was found to be significantly upregulated in the liver of rats with HE [21]. After NF-*κ*B activation, inflammatory factors released can in turn further activate NF-*κ*B and amplify the inflammatory response cascade, thus generating a vicious cycle that would eventually lead to massive hepatocyte necrosis. Consequently, the synthesis, metabolism, and detoxification functions of the liver would be hampered and excessive ammonia and endotoxin that cannot be neutralized by the liver would enter blood circulation. Hyperammonemia can stimulate the expression of nitric oxide synthase (iNOS), upregulate the production of nitric oxide (NO), and increase cerebral blood flow, thus leading to edema of astrocytes and damage to the central nervous system [45], which ultimately causes cognitive dysfunction. On the other hand, inflammatory cytokines released after NF-*κ*B activation can enter the peripheral blood circulation to aggravate infection and induce systemic inflammatory response, thereby playing an important role during pathogenesis and progression of HE synergistically with hyperammonemia [46]. In short, the NF-*κ*B signaling pathway triggers the release of inflammatory factors, amplifies liver inflammatory response, accelerates liver function damage, and thereby contributes to the pathogenesis of HE. Mitigating inflammation, both systematically and locally in the liver, can potentially alleviate the severity of HE. In this study, we evaluated the role of EA treatment in an established rat HE model and found that EA therapy reduced IL-1*β*, IL-6, and TNF-*α* levels in the hippocampus, and combination of EA and drugs significantly downregulated mRNA and protein expressions of iNOS, TLR4, MyD88, and NF-*κ*B. Compared with the CCl_4_ + Lac group, the CCl_4_ + EA and CCl_4_ + CM groups had significant effects. Because EA and lactulose are both effective treatment methods, the combination of EA and lactulose has the best effect. Based on findings that the TLR4/MyD88/NF-*κ*B signaling pathway plays an important role in mediating inflammatory response and that EA can inhibit inflammatory response through the NF-*κ*B signaling pathway, we speculate that EA may inhibit intracerebral inflammatory response through the TLR4/MyD88/NF-*κ*B signaling pathway, thereby improving the cognitive dysfunction in HE.

The article "Electroacupuncture Synergistically Inhibits Proinflammatory Cytokine Production and Improves Cognitive Function in Rats with Cognitive Impairment due to Hepatic Encephalopathy through p38MAPK/STAT3 and TLR4/NF-κB Signaling Pathways" was published in 2021. Journal: Evid Based Complement Alternat Med.

The P38MAPK signaling pathway is an important member of the mitogen-activated protein kinase family, which can be activated by a variety of stress stimuli including reactive oxygen species and plays an important role in processes such as inflammatory response, cellular stress response, and cell apoptosis. Studies have reported that signaling pathways including p38MAPK play an important role in the pathogenesis and treatment of HE [47] and that inhibition of MAPKs can improve the cognitive function in animal models of HE. Activation of p38 and JNKMAPKs in astrocytes may lead to astrocyte swelling that affects glutamate uptake [48]. P38MAPK also plays anti-inflammatory and antioxidative roles via mediating the STAT3 pathway [49] through direct phosphorylation of the serine residues at the STAT3-C terminal, and STAT3 is therefore considered one of the possible substrates of MAPK. Under certain stimulating factors (such as inflammation and oxidative stress), MAPK and STAT3 signaling pathways may be concomitantly activated [50]. In this study, compared with the CCl_4_ group, the mRNA and protein expressions of p38MAPK, p-p38MAPK, STAT3, and p-STAT3 in brain tissues of HE rats in all treatment groups were significantly decreased (*P* < 0.05). Compared with the CCl_4_ + Lac group, expressions of p38MAPK, p-p38MAPK, STAT3, and p-STAT3 in the CCl_4_ +CM group were significantly downregulated. Thus, the p38MAPK-STAT3 signaling pathway was found to be activated. EA treatment mitigated the phosphorylation of p38MAPK and STAT3 induced by combined treatment with CCl_4_ and thioacetamide and downregulated the expressions of p38MAPK and STAT3 mRNAs, as well as their phosphorylated proteins. Additionally, pathologic injury to the liver in rats with HE was alleviated by EA therapy. These results suggest that the p38MAPK-STAT3 signaling pathway is involved in the regulation of HE and EA may play anti-inflammatory and antioxidative roles through regulating the p38MAPK-STAT3 signaling pathway, thus improving the cognitive impairment in HE.

The article "Electroacupuncture Synergistically Inhibits Proinflammatory Cytokine Production and Improves Cognitive Function in Rats with Cognitive Impairment due to Hepatic Encephalopathy through p38MAPK/STAT3 and TLR4/NF-κB Signaling Pathways" was published in 2021. Journal: Evid Based Complement Alternat Med.

In addition, as for the relationship among MRS, serum ammonia, liver function markers, and the expressions of certain genes and proteins in the brain tissue, the expressions of TNF-*α*, IL-1*β*, IL-6, and TLR4 were positively correlated with serum ammonia concentration in hepatic encephalopathy model rats. Serum ammonia and inflammatory mediators synergistically affect the occurrence and development of HE through Pearson's correlation analysis and literature review. Ammonia is a neurotoxin that leads to a variety of neurological complications, and it causes oxidative stress and brain edema and triggers neuroinflammation [51]. Inflammation is central to the pathogenesis of many human neurological disorders including HE. Systemic inflammation is a key player in precipitating and exacerbating HE, possibly by rendering the brain more susceptible to concurrent hyperammonemia [52]. Activated microglia also release proinflammatory mediators (e.g., cytokines TNF-*α*, IL-6, and IL-1*β*) that have also been directly linked to brain dysfunction [45]. It has been previously reported that activation of TLR4 initiates the NF-*κ*B pathway as it stimulates the expression of proinflammatory cytokines TNF-*α*, IL-6, and IL-1*β*, which finally contributes to astrocyte swelling in HE [53]. MRS reflects the changes of brain metabolites such as mIns and Glx in the diagnosis of hepatic encephalopathy. Studies by Kooka et al. have shown that serum ammonia levels are negatively correlated with Cho and mIns levels in MRS and positively correlated with Glx levels [39]. Brain Glx levels are significantly positively correlated with serum TNF-*α* and IL-6 levels. The increase of TNF-*α* and IL-6 levels may increase the accumulation of Glx in astrocytes and promote the occurrence of cerebral edema. HE staining reflects the changes of astrocytes and neurons in the brain tissue. This experiment also shows that EA has a neuroprotective effect and can improve brain injury. AST, TBil, ALT, etc., are all typical biochemical test indicators, which can effectively reflect the inflammatory state of the liver and the degree of tissue cell damage. The correlation analysis shows that serum TNF-*α*, IL-6, and IL-1*β* levels are not significantly correlated with liver function indexes such as AST, ALT, TBil, and ALB. The reason may be due to the small sample size, a lot of experimental research is still needed in the future.

The article "Electroacupuncture Synergistically Inhibits Proinflammatory Cytokine Production and Improves Cognitive Function in Rats with Cognitive Impairment due to Hepatic Encephalopathy through p38MAPK/STAT3 and TLR4/NF-κB Signaling Pathways" was published in 2021. Journal: Evid Based Complement Alternat Med.

## 5. Conclusions

In conclusion, the synergistic role of inflammation and hyperammonemia can further aggravate the impaired cognitive function in HE. Treatment with EA may reduce the blood ammonia level, modulate inflammatory factors, ameliorate brain necrosis and apoptosis, and improve cognitive impairment through regulation of TLR4/MyD88/NF-*κ*B and p38MAPK/STAT3 signaling pathways. MRS may be valuable in HE diagnosis of and evaluation of acupuncture efficacy. There are some limitations in the scope of this study, which are relatively simple compared with the complicated pathogenesis of HE involving multiple inflammatory reaction pathways. Future studies should adopt multimodal function imaging techniques, expand the sample size, and design rigorous experimental approaches to further explore the mechanism of acupuncture in improving cognitive dysfunction in HE.

## Figures and Tables

**Figure 1:** Wistar rats were treated with intraperitoneal injections of 1 mL/kg of 35% CCl_4_ twice a week for 9 weeks. When liver cirrhosis models were established, rats with cognitive impairment were screened through the Morris water maze test and randomly divided into a no-intervention group (CCl_4_) and treatment groups including EA group (CCl_4_ + EA), lactulose group (CCl_4_ + Lac), and EA combined with lactulose group (CCl_4_ + CM), with 9 rats in each group. Ten rats in the normal group. (a–c) Behavior trajectory of rats before modeling, after modeling, and after treatment; (d) escape latency; and (e) times of crossing the platform. ^#^*P* < 0.05 versus normal group. ^*∗*^*P* < 0.05 versus CCl_4_ model group.

**Figure 2:** Wistar rats were treated with intraperitoneal injections of 1 mL/kg of 35% CCl_4_ twice a week for 9 weeks. When liver cirrhosis models were established, rats with cognitive impairment were screened through the Morris water maze test and randomly divided into a no-intervention group (CCl_4_) and treatment groups including EA group (CCl_4_ + EA), lactulose group (CCl_4_ + Lac), and EA combined with lactulose group (CCl_4_ + CM), with 9 rats in each group. There are 10 rats in the normal group. (a–g) Serum levels of ALT, AST, TBA, TBil, TP, ALB, and blood ammonia. The results are expressed as mean ± SD. ^###^*P* < 0.001 and ^##^*P* < 0.01 versus normal group.  ^*∗*^*P* < 0.05,  ^*∗*^ ^*∗*^*P* < 0.01, and  ^*∗*^ ^*∗*^ ^*∗*^*P* < 0.001 versus CCl_4_ model group. ALT: alanine aminotransferase; AST: aspartate aminotransferase; TBA: total bile acid; TBil: total bilirubin; TP: total protein; ALB: albumin.

**Figure 3:** EA improved the brain injury induced by CCl_4_ combined with TAA in HE rats.

The article "Electroacupuncture Synergistically Inhibits Proinflammatory Cytokine Production and Improves Cognitive Function in Rats with Cognitive Impairment due to Hepatic Encephalopathy through p38MAPK/STAT3 and TLR4/NF-κB Signaling Pathways" was published in 2021. Journal: Evid Based Complement Alternat Med.

**Figure 4:** There are 10 rats in the normal group and 9 rats in each of no-intervention group (CCl_4_) and treatment groups including EA group (CCl_4_ + EA), lactulose group (CCl_4_ + Lac), and EA combined with lactulose (CCl_4_ + CM) group. (a) MRS map. (b) Comparison of the subpeak area ratio of metabolites in the brain tissue of five groups. The results are expressed as mean ± SD. ^###^*P* < 0.001 versus normal group.  ^*∗*^*P* < 0.05,  ^*∗*^ ^*∗*^*P* < 0.01, and  ^*∗*^ ^*∗*^ ^*∗*^*P* < 0.001 versus CCl_4_ model group.

**Figure 5:** Wistar rats were treated with intraperitoneal injections of 1 mL/kg of 35% CCl_4_ twice a week for 9 weeks. When HE models were established, the lactulose group (CCl_4_ + Lac) and acupuncture combined with medicine group (CCl_4_ + CM) were gavaged with 10 mL/kg body weight. EA was given to the EA (CCl_4_ + EA) and the combination (CCl_4_ + CM) groups 30 min per day with consecutive 21 days. There are 10 rats in the normal group, and 9 rats in each of no-intervention group (CCl_4_) and treatment groups including EA group (CCl_4_ + EA), lactulose group (CCl_4_ + Lac), and EA combined with lactulose (CCl_4_ + CM) group. Expressions of TNF-*α*, IL-6, IL-1*β*, iNOS, TLR4, MyD88, NF-*κ*B, p38MAPK, and STAT3 genes were used to evaluate hepatic inflammation in the mRNA level detected by RT-qPCR.

**Figure 6:** EA regulates the expression level of hepatic inflammation pathway-related proteins. There are 10 rats in the normal group and 9 rats in each of no-intervention group (CCl_4_) and treatment groups including EA group (CCl_4_ + EA), lactulose group (CCl_4_ + Lac), and EA combined with lactulose (CCl_4_ + CM) group. (a–i) TNF-*α*, IL-6, TLR4, MyD88, NF-*κ*B, p38MAPK, p-p38MAPK, STAT3, and p-STST3 were used to evaluate the degree of inflammation in protein levels detected by Western blot. ^###^*P* < 0.001 versus normal group.  ^*∗*^*P* < 0.05,  ^*∗*^ ^*∗*^*P* < 0.01, and  ^*∗*^ ^*∗*^ ^*∗*^*P* < 0.001 versus CCl_4_ model group.

**Figure 7:** EA regulates the expression level of hepatic inflammation pathway-related proteins detected by Western blot. There are 10 rats in the normal group and 9 rats in each of no-intervention group (CCl_4_) and treatment groups including EA group (CCl_4_ + EA), lactulose group (CCl_4_ + Lac), and EA combined with lactulose (CCl_4_ + CM) group. (a) The protein expression of TNF-*α* and IL-6. (b) TLR4 pathway-associated signal proteins TLR4, MyD88, and NF-*κ*B. (c) Proteins expressions of phosphorylated and total p38MAPK and STAT3.

**Table 1:** Sequences of primers used in real-time polymerase chain reactions.

Genes	Sequences of primers	GenBank accession number	Annealing Tm (°C)	Product size (bp)
iNOS	5′CTTGGAGCGAGTTGTGGATTGT3′	NM_012611.3	60	148
	5′GGTAGTGATGTCCAGGAAGTAGGTG 3′			

TNF-*α*	5′CCACCACGCTCTTCTGTCTACTG3′	NM_012675.3	60	151
	5′ TGGGCTACGGGCTTGTCACT 3′			

IL-1*β*	5′CTGTGACTCGTGGGATGATGA3′	NM_031512.2	60	161
	5′ CCACTTGTTGGCTTATGTTCTGTC 3′			

IL-6	5′CAGCGATGATGCACTGTCAGA3′	NM_012589.2	60	287
	5′ GGAGAGCATTGGAAGTTGGGG 3′			

TLR4	5′AGCCTTGAATCCAGATGAAAC3′	NM_019078	60	135
	5′ ACAGCAGAAACCCAGATGAA 3′			

MyD88	5′TCCAACAGAAGCGACTGAT3′	NM_198130	60	83
	5′ GCAGATAGTGATGAACCGTAG 3′			

NF-*κ*B	5′GCTCCTTTTCTCAAGCCGATGT3′	NM_199267.2	60	145
	5′ CGTAGGTCCTTTTGCGTTTTTC 3′			

P38MAPK	5′TGTGATTGGTCTGTTGGATGTGT3′	NM_031020.2	60	200
	5′ TGTGGATTATGTCAGCCGAGTG3′			

STAT3	5′GCCATCCTAAGCACAAAGCC3′ 5′GGGAATGTCAGGGTAGAGGTAGA3′	NM_012747.2	60	249

*β*-Actin	5′CCTCTATGCCAACACAGT3′	NM_031144	60	155
	5′ AGCCACCAATCCACACAG 3′			

The article "Electroacupuncture Synergistically Inhibits Proinflammatory Cytokine Production and Improves Cognitive Function in Rats with Cognitive Impairment due to Hepatic Encephalopathy through p38MAPK/STAT3 and TLR4/NF-κB Signaling Pathways" was published in 2021. Journal: Evid Based Complement Alternat Med.

## Data Availability

The data used to support the findings of this study are available from the corresponding author upon request.
